The article "LncRNA SNHG10 suppresses the development of doxorubicin resistance by downregulating miR-302b in triple-negative breast cancer" was retracted in 2026. Reasons: concerns about the data; concerns about the results or conclusions.

# LncRNA SNHG10 suppresses the development of doxorubicin resistance by downregulating miR-302b in triple-negative breast cancer

**DOI:** 10.1080/21655979.2022.2063592

**Published:** 2022-05-03

**Authors:** Shataer Aini, Shayiti Bolati, Wei Ding, Siyin Liu, Pengcheng Su, Saiding Aili, Yimin Naman, Kuerban Xuekelaiti

**Affiliations:** Department of Mammary Gland and Thyroid Surgery, People’s Hospital of Xinjiang Uygur Autonomous Region, Urumqi, Xinjiang, China

**Keywords:** SNHG10, triple negative breast cancer, doxorubicin, miR-302b, apoptosis

## Abstract

Unlike other types of breast cancer, triple negative breast cancer (TNBC) does not respond to therapies targeting human epidermal growth factor receptor-2 (HER2) or hormone therapy, and the prognosis of patients with TNBC is usually poor. The role of long non-coding RNA (lncRNA) small nucleolar RNA host gene 10 (SNHG10) has been investigated in many types of cancer, but its role in TNBC is unknown. This study aimed to explore the role of SNHG10 in TNBC in the context of doxorubicin treatment, a common therapy for TNBC. Analysis of the TCGA dataset revealed the downregulation of SNHG10 in TNBC. The downregulation of SNHG10 of TNBC in TNBC was further confirmed by detecting its expression in 60 patients with TNBC by qPCR. The expression of SNHG10 was further downregulated after doxorubicin treatment. In TNBC, microRNA-302b (miR-302b) was downregulated and was positively correlated with SNHG10. In TNBC cells, overexpression of SNHG10 resulted in upregulation of miR-302b, and methylation-specific PCR analysis showed that SNHG10 negatively regulates the methylation of miR-302b. In addition, doxorubicin treatment resulted in the downregulation of SNHG10 in TNBC cells, and overexpression of SNHG10 and miR-302b promoted apoptosis of doxorubicin-treated TNBC cells. Furthermore, overexpression of both SNHG10 and miR-302b had a stronger effect on apoptosis than that of overexpression of SNHG10 alone. Our study showed that SNHG10 could inhibit the development of resistance to doxorubicin by upregulating miR-302b in TNBC through methylation. Our findings suggested that SNHG10 might serve as a molecular target for intervening in TBNC metastasis.

## Highlights

- MiR-302b expression was positively correlated with SNHG10.
- Overexpression of SNHG10 upregulates miR-302b
- SNHG10 negatively regulates the methylation miR-302b.
- Overexpression of SNHG10 and miR-302b promoted apoptosis of doxorubicin-treated TNBC cells.
- Overexpression of both SNHG10 and miR-302b had a stronger effect on apoptosis than overexpression of SNHG10 alone.

## Introduction

In 2018, breast cancer accounted for 11.6% of newly diagnosed cancers [1]. Triple-negative breast cancer (TNBC), which is negative for HER2 and estrogen and progesterone receptors, is a common subtype of breast cancer [2]. Unlike other types of breast cancer, TNBC does not respond to HER2-targeting or hormonal therapies [3]. Therefore, the prognosis of patients with TNBC is generally poor. The 5-year survival rate of early TNBC and advanced TNBC is about 77% and 14%, respectively [4]. Drugs, such as doxorubicin, are commonly used to treat TNBC. However, chemoresistance often develops, and the long-term treatment outcomes are poor [5].

Previous studies have identified various molecules involved in the development of resistance in TNBC cells to doxorubicin, such as 5’-nucleotidase, ecto (CD73) and hypoxia-induced tRNA-derived fragments [6,7]. In addition, a considerable number of long non-coding RNAs (lncRNAs) have been shown to regulate the expression of cancer-related genes in nearly all aspects of cancer biology [8,9], including chemoresistance [10]. Therefore, regulating the expression of certain lncRNAs may increase the drug sensitivity of cancer cells [11]. However, the functions of most lncRNAs in cancer biology remain unclear.

Several small nucleolar RNA host genes (SNHGs) have been identified as key factors in carcinogenesis and metastasis. For example, lncRNA SNHG10 was recently identified as a oncogene in liver cancer [12], and small nucleolar RNA host gene 6 (SNHG6) was shown to regulate the overall DNA methylation levels by activating the miR-1297/FUS pathway, which inhibits the expression of MAT1A, thereby promoting the phenotype of liver cancer cells. Small nucleolar RNA host gene 15 (SNHG15) maintains the stability of Slug in colon cancer cells by interacting with its zinc finger domain, which promotes the migration of colon cancer cells [13]. SNHG10 was highly expressed in 64 HCC tissues and predicted poor survival of patients [12]. In contrast, analysis of TCGA dataset revealed the downregulation of SNHG10 in TNBC. Therefore, SNHG10 may play different roles in different types of cancer.

MicroRNAs (miRNAs) play vital roles in breast cancer. miR-302b was downregulated in breast cancer (BC) [14]. Moreover, the expression of miR-302b predicts the mortality rate of patients [15]. From our preliminary sequencing analysis, we observed that SNHG10 and miR-302b were closely correlated, and miR-302b plays a critical role in regulating the sensitivity of TNBC cells to chemotherapy [15]. Therefore, we hypothesized that SNHG10 and miR-302b may interact with each other to participate in TNBC. The role of SNHG10 has been investigated in many types of cancer, but its role in TNBC is unknown. This study aimed to explore the role of SNHG10 in TNBC in the context of doxorubicin treatment, a common therapy for TNBC. Our findings showed that SNHG10 could inhibit the development of resistance to doxorubicin by upregulating miR-302b in TNBC through methylation.

## Materials and methods

### Triple negative breast cancer (TNBC) patients

This study included 60 TNBC patients (all females, 38–66 years old; mean age, 47.9 ± 4.9 years old) who were admitted to People’s Hospital of Xinjiang Uygur Autonomous Region from May 2017 through May 2019. This study was approved by the Ethics Committee of this hospital. All patients with TNBC were diagnosed for the first time. Patients with a family history or previous history of malignancy were excluded. Patients who had initiated therapy were excluded. Written informed consent was obtained from all patients.

### Treatment and specimen collection

The study group of 60 patients included 28 patients with AJCC stage II disease and 32 patients with stage III disease. All patients were treated with four courses of doxorubicin (25,316–40-9; Sangon Biotech) at a dose of 100 mg/m^2^ and 21 days per course. TNBC tissues and adjacent (within 3 cm of the tumor) normal tissues were collected. FNA biopsy was also performed on all patients after treatment to collect TNBC tissues.

### Triple negative breast cancer (TNBC) cells

TNBC cell lines BT-549 and MDA-MB-157 (ATCC) were used. The cells were cultivated in RPMI-1640 culture medium (11,875,101, Thermo Fisher) containing 10% fetal bovine serum (FBS, sh30370.03, Beijing Formula Biological Co., Ltd., China) in a 5% CO_2_ incubator at 37°C and 95% humidity. Cells were collected at approximately 80% confluence for subsequent experiments [16].

### Cell transfections

BT-549 and MDA-MB-157 cells were collected and counted, and then 10^6^ cells were transfected with SNHG10 vector (pcDNA3.1, kl-zl-0650, Shanghai Kelei Biotechnology Co., Ltd., China) and/or miR-302b mimic (miRA1000925-1-100, Guangzhou Ribo Biological Co., Ltd., China) for 6 h using Lipofectamine 2000 reagent. Cells transfected with NC miRNA or an empty vector were used as negative controls (NC). Cells were harvested after 48 h for subsequent experiments [17].

### RNA extraction and Reverse Transcription-Polymerase Chain Reaction (RT-qPCR)

Total RNAs were isolated from both tissues and cells using RNAzol reagent (RTN70, Sigma-Aldrich) [18]. Cells were treated with doxorubicin at doses of 0, 1, 5, and 10 ng/ml for 48 h before RNA isolation. The Bio-Rad iScript cDNA Synthesis Kit (170–8891, Bio-Rad, America) was used to synthesize cDNA from the extracted RNA. The KAPA SYBR® FAST qPCR Master Mix Kit (KK4606, KAPA, America) was used for all qPCR reactions using the synthesized cDNA as templates with glyceraldehyde-3-phosphate dehydrogenase (GAPDH) as the internal control. The All-in-One™ miRNA qRT-PCR Detection Kit (QP115, Genecopoeia) was used to generate mature miRNA poly (A), to reverse transcribe the miRNAs, and to perform qPCR reactions [19]. The expression of miR-302b was measured using U6 as the internal control. The 2^−ΔΔCT^ method was used to calculate the fold changes in expression levels. The primer sequences are shown in Table S1.

### Methylation-specific Polymerase Chain Reaction (PCR)

Genomic DNA was isolated from *in vitro* cultured cells using the Genomic DNA Extraction Kit (ab156900; Abcam). The DNA Methylation-Gold^TM^ kit (D5006, Zymo Research) was used for bisulfite-conversion of genomic DNA. Methylation-specific PCR (MSP) was then performed using a Taq DNA polymerase kit (201,203, Shanghai QIAGEN Biological Co., Ltd., China) to assess the methylation of miR-302b gene [20].

### Cell apoptosis assay

Apoptosis of BT-549 and MDA-MB-157 cells was assessed at 48 h after transfection and incubation with medium containing 10 ng/ml doxorubicin for another 48 h. The cells were then washed twice with cold PBS and centrifuged. Then, the pellets, containing 10^6^ cells, were stained with both FITC-labeled Annexin-V (5 µL) and PI solution (5 µL) for 20 min in the dark. Finally, apoptotic cells were separated and enumerated using flow cytometry [21].

### Cell proliferation assay

BT-549 cells were seeded in a 96-well plate (2 × 10^3^/well) at 0, 24, 48, and 72 h after transfection, and cell proliferation was assessed using the counting kit-8 (CCK-8) and colony formation assay. The CCK-8 assay was performed using a commercial kit (CK04-11, Dojindo Laboratories, Dojindo, Japan). The colony formation assay was performed as previously described [22].

### Transwell assay

Transfected BT-549 cells (5 × 10^4^) were suspended in 200 μL of serum-free medium and seeded in the upper chamber of a Transwell insert (3413, Beijing Borunlaite Science and Technology Co., Ltd, China) [23]. Cell movement was analyzed as previously described.

### Statistical analysis

Data were expressed as the mean values of three biological replicates. A paired t-test was used to compare the two types of tissue samples and the two time points (pre- and post-treatment). Correlations were analyzed by linear regression. ANOVA and Tukey’s test were used to compare multiple groups. Statistical significance was set at *P* < 0.05.

## Results

The role of SNHG10 has been investigated in many types of cancer, but its role in TNBC is unknown. This study aimed to explore the role of the SNHG10 in TNBC in the context of doxorubicin treatment, a common therapy for TNBC. Analysis of the TCGA dataset and qPCR revealed the downregulation of SNHG10 in TNBC. In TNBC, miR-302b was downregulated and was positively correlated with SNHG10. In TNBC cells, overexpression of SNHG10 resulted in upregulation of miR-302b, and the methylation-specific PCR analysis showed that SNHG10 negatively regulates the methylation miR-302b. Doxorubicin treatment resulted in the downregulation of SNHG10 in TNBC cells, and overexpression of SNHG10 and miR-302b promoted apoptosis of doxorubicin-treated TNBC cells. In addition, overexpression of both SNHG10 and miR-302b had a stronger effect on apoptosis than overexpression of SNHG10 alone. Our study showed that SNHG10 could inhibit the development of resistance to doxorubicin by upregulating miR-302b in TNBC through methylation.

### Small nucleolar RNA host gene 10 (SNHG10) was downregulated in triple negative breast cancer (TNBC) and was further downregulated by doxorubicin treatment

The expression of SNHG10 was analyzed in a TNBC dataset from TCGA using Gepia (http://gepia.cancer-pku.cn/detail.php?gene=SNHG10). The analysis showed that the expression levels of SNHG10 were lower in TNBC tissues than that in non-tumor tissues (4.98 vs. 7.62 reads per million). To confirm this finding, the expression levels of SNHG10 were measured in TNBC tissues and adjacent non-tumor tissues collected from 60 patients with TNBC by RT-qPCR. It was observed that SNHG10 was downregulated in TNBC tissues compared to that in non-tumor tissues (Figure 1, p < 0.0001). The expression levels of SNHG10 in TNBC tissues were also measured by RT-qPCR after doxorubicin treatment. Compared to pre-treatment levels, the expression levels of SNHG10 were significantly lower after treatment (Figure 1, p < 0.05). Therefore, downregulation of SNHG10 may participate in TNBC and doxorubicin treatment.

**Figure 1.** **SNHG10 is downregulated in triple-negative breast cancer and is further downregulated by doxorubicin treatment**. The expression levels of SNHG10 in triple-negative breast cancer (TNBC) tissues and adjacent non-tumor tissues before treatment were measured by RT-qPCR. The expression levels of SNHG10 in TNBC tissues were also measured by RT-qPCR after doxorubicin treatment. All reactions were performed in triplicate, and a paired t test was used to compare the mean values between the two tissue types and two time points. *, *p* < 0.05; ***, *p* < 0.001.

### MiR-302b was downregulated in triple negative breast cancer (TNBC) and was positively correlated with small nucleolar RNA host gene 10 (SNHG10) levels

Expression of miR-302b in paired tissues from 60 patients with TNBC was also analyzed using RT-qPCR. RT-qPCR analysis revealed significantly lower expression levels of miR-302b in TNBC tissues compared to that in non-tumor tissues (Figure 2(a), p < 0.0001). The correlation of SNHG10 to miR-302b was analyzed using Pearson’s correlation coefficient. SNHG10 and miR-302b were significantly, positively correlated across TNBC tissues (Figure 2(b)) and non-tumor tissues (Figure 2(c)).

**Figure 2.** **MiR-302b is downregulated in TNBC and is positively correlated with SNHG10**. The expression levels of miR-302b in both TNBC and adjacent non-tumor tissues were measured by RT-qPCR. All reactions were performed in triplicate, and a paired t test was used to compare the mean values between the two types of tissues (a). ***, *p* < 0.001. Correlations between the expression levels of SNHG10 and miR-302b in TNBC tissues (b) and non-tumor tissues (c) were analyzed by linear regression.

### Small nucleolar RNA host gene 10 (SNHG10) upregulated miR-302b through methylation

The close correlation between SNHG10 and miR-302b indicated a possible interaction between them. To explore their interaction, BT-549 and MDA-MB-157 cells were transfected with a miR-302b mimic or SNHG10 expression vector, and overexpression of miR-302b and SNHG10 were confirmed by RT-qPCR at 48 h after transfection (Figure 3(a), p < 0.05). Compared to control and NC miRNA transfected cells, no alteration in the expression levels of SNHG10 was observed in cells transfected with miR-302b mimic, suggesting that miR-302b did not regulate the expression of SNHG10 (Figure 3(b)). However, overexpression of SNHG10 resulted in the upregulation of miR-302b (Figure 3(c), p < 0.05). MSP was performed to evaluate the effect of overexpression of SNHG10 on miR-302b gene methylation, and the results showed that SNHG10 suppressed miR-302b gene methylation (Figure 3(d), p < 0.05).

**Figure 3.** **SNHG10 upregulates miR-302b levels through methylation**. BT-549 and MDA-MB-157 cells were transfected with either a miR-302b mimic or SNHG10 expression vector, and overexpression was confirmed by RT-qPCR 48 h later (a). The effects of miR-302b overexpression on the expression of SNHG10 (b) and the effects of SNHG10 overexpression on miR-302b (c) were also analyzed by RT-qPCR. Methylation-specific PCR analysis of the miR-302b gene. U refers to the U6 control, and M refers to miR-302b. (d). *, *p* < 0.05.

### Small nucleolar RNA host gene 10 (SNHG10) and miR-302b promoted doxorubicin-induced apoptosis of triple negative breast cancer (TNBC) cells

BT-549 and MDA-MB-157 cells were treated with doxorubicin at doses of 0, 1, 5, and 10 ng/ml for 48 h, and the expression levels of SNHG10 were measured using RT-qPCR. Doxorubicin treatment decreased the expression levels of SNHG10 in TNBC cells (Figure 4(a), p < 0.05). The role of SNHG10 and miR-20b in the apoptosis of BT-549 and MDA-MB-157 cells was analyzed. Overexpression of SNHG10 and miR-302b promoted the apoptosis of TNBC cells with doxorubicin treatment (Figure 4(b), p < 0.05). In addition, overexpression of both SNHG10 and miR-302b showed a much stronger effect on doxorubicin-induced cell apoptosis (*p* < 0.05).

**Figure 4.** **SNHG10 and miR-302b promote doxorubicin-induced TNBC cell apoptosis**. BT-549 and MDA-MB-157 cells were treated with doxorubicin at doses of 0, 1, 5 and 10 ng/ml for 48 h, and then the expression levels of SNHG10 were measured using RT-qPCR (a). A cell apoptosis assay was performed to analyze the effects of overexpression of SNHG10 and miR-20b on the apoptosis of BT-549 and MDA-MB-157 cells (b). *, *p* < 0.05.

Furthermore, CCK-8 assay was performed to evaluate the proliferation of BT-549 cells transfected with SNHG10 vector or co-transfected with SNHG10 and miR-302b mimic (Figure 5(a), p < 0.05). Colony formation assay was used to evaluate the proliferation of TNBC cells transfected with SNHG10 or co-transfected with SNHG10 and a miR-320b mimic (Figure 5(b), p < 0.05). It was observed that SNHG10 suppressed cell proliferation and colony formation, The addition of miR-320b enhanced the inhibitory effects.

**Figure 5.** **SNHG10 and miR-302b regulates the proliferation and colony formation of BT-549 cell apoptosis**. The proliferation (a) and colony formation of BC cells transfected with SNHG10 or co-transfected with SNHG10 and a miR-302b mimic was evaluated using the CCK-8 assay and colony formation assay, respectively. Colony formation assay (b) was used to evaluate the proliferation of TNBC cells transfected with SNHG10 or co-transfected with SNHG10 and a miR-320b mimic. **, *p* < 0.01.

## Discussion

The morbidity and mortality of breast cancer rates are expected to increase significantly in the near future [24]. TNBC accounts for approximately 20% of all breast cancers. The management of TNBC is challenging due to its aggressive phenotype, heterogeneity, and lack of targeted therapy [25]. TNBC is an orphan disease for which treatment has not progressed in the past a few decades, and the standard treatment is still chemotherapy [26]. We in this study aimed to explore possible molecular players in TNBC. The characterized critical molecular players in TNBC may serve as potential targets to treat TNBC.

In recent years, gene therapy has become a research hotspot. LncRNAs are involved in the regulation of various intracellular processes, and are closely related to the occurrence and development of various tumors, and therefore are considered to be new targets for the treatment of distant metastases in breast cancer. LncRNA H19 has been confirmed to be involved in many biological processes in various tumors, such as tumor cell proliferation, invasion and apoptosis. In breast cancer, abnormal expression of H19 may be related to tumor epidermal growth factor receptor 2 (HER2) positivity. In an *in vitro* experimental model, H19 can stimulate the proliferation of breast cancer cells and inhibit apoptosis [27]. LncRNAs can regulate the occurrence and development of breast cancer at different levels, such as the transcriptional level or the post-transcriptional level. Different lncRNA-involved pathways might serve as new targets for breast cancer treatment in the future. However, the mechanisms underlying the regulation of most lncRNAs in breast cancer are still unclear.

SNHG10 was recently shown to play an oncogenic role in liver cancer [12]. SNHG10 was also shown to be a predictor of poor survival in patients with liver cancer [28]. In addition, SNHG10 regulates the expression of its homolog SCARNA13 to promote tumor metastasis [12,29]. To date, little is known about the biological role of SNHG10 in TNBC. In this study, we analyzed a TNBC dataset in TCGA and observed downregulation of SNHG10 in TNBC. We also measured the expression levels of SNHG10 in 60 sets of paired TNBC [30] and adjacent non-tumor tissues from patients with TNBC and observed downregulation of SNHG10 in the TNBC tissues. Moreover, overexpression of SNHG10 increased the sensitivity of TNBC cells to doxorubicin, suggesting that SNHG10 likely functions as a tumor suppressor in TNBC. Therefore, this lncRNA may play different roles in different types of cancer.

A recent study reported that overexpression of miR-302b enhanced the sensitivity of breast cancer cells to cisplatin by regulating the cellular DNA damage response and the expression of E2F1 [31]. In this study, we showed that overexpression of miR-302b also increased the sensitivity of TNBC cells to doxorubicin. Interestingly, our study showed that SNHG10 upregulated the expression of miR-302b. It has been reported that lncRNAs can regulate the expression of miRNAs through methylation pathways [32]. For instance, the lncRNA PVT1 downregulated miR-146a by increasing the methylation level of the miR-146a gene to regulate tumor growth in prostate cancer [33]. Our study is the first to report the regulation of miR-302b expression by a lncRNA through methylation. However, our study only reported that SNHG10 decreased the methylation level of the miR-302b gene in TNBC cells, but the molecular mechanism is not yet known. In this study, we explored the interaction between SNHG10 and miR-302b in TNBC and found that the expression levels of SNHG10 and miR-302b were altered in TNBC cells. Therefore, altered expression of SNHG10 in TNBC cells may upregulate miR-302b to increase the sensitivity of TNBC cells to doxorubicin. Interestingly, SNHG10 and miR-302b were closely correlated across TNBC and non-tumor tissues, suggesting that they may interact with each other under both pathological and physiological conditions. However, altered expression of SNHG10 and miR-302b was observed in TNBC. We speculated that it is the altered expression, but not the interaction alone, drives the progression of TNBC.

## Conclusion

In conclusion, this study demonstrated that SNHG10 and miR-302b are downregulated in TNBC [34,35]. Overexpression of SNHG10 may serve as a potential target to treat TNBC by upregulating miR-302b through methylation, thereby increasing the sensitivity of TNBC cells to doxorubicin.

## Supplementary Material

Supplemental Material

## Data Availability

The datasets used and analyzed during the current study are available from the corresponding author upon reasonable request.
